The article "Associated Factors of Wasting among Infants and Young Children (IYC) in Kuyu District, Northern Oromia, Ethiopia" was published in 2022. Journal: Biomed Res Int.

# Associated Factors of Wasting among Infants and Young Children (IYC) in Kuyu District, Northern Oromia, Ethiopia

**DOI:** 10.1155/2022/9170322

**Published:** 2022-06-30

**Authors:** Tamiru Yazew, Agama Daba

**Affiliations:** Department of Food and Nutritional Sciences, Wollega University, Shambu, Ethiopia

## Abstract

Wasting among infants and young children in underdeveloped countries including Ethiopia is one of the most serious public health issues. Therefore, this study was designed to assess the magnitude of wasting and the variables that associate with it among infants and young children in the Kuyu district of Northern Oromia, Ethiopia. A community-based cross-sectional study of 612 infants and young children aged 6-23 months was conducted. To select eligible infants and young children from each family in the Kuyu district, a multilevel sampling approach was used. The amount and determinants related to wasting were investigated using the Statistical Package for Social Sciences (SPSS) version 20.0. In the study area, 14.1% of infants and young children were found to be wasting. Maternal educational status (AOR = 1.8, 95% CI; 1.01, 4.32), diarrhoea (AOR = 2.3, 95% CI; 1.98, 4.56), exclusive breastfeeding (AOR = 2.46, 95% CI, 1.4, 4.58), antenatal care visits (AOR = 2.21; 95% CI, 1.32, 3.48), and wealth index (AOR = 1.66, 95% CI; 1.07, 4.47) were significantly associated with wasting. According to the findings of this study, mother educational status, the occurrence of diarrhoea, exclusive breastfeeding, antenatal care visits, and wealth index have an impact on infants and young children's wasting. Therefore, to lower the burden of wasting among infants and young children in the study, community-based schooling and nutritional interventions are urgently needed.

## 1. Introduction

Wasting is one of the world's most difficult issues, affecting mostly underprivileged and disadvantaged areas [1], and it causes disease and mortality in infants and young children [2]. Its high occurrence has been shown to have negative consequences on a child's survival, growth, and cognitive development [3]. In developing countries, it is a well-known indicator of infant and young child nutrition [4]. Worldwide, 51 million infants and young children are expected to be underweight for their height [5]. This prevalence was estimated to be 12.9%, with almost 90% of people residing in low- and middle-income countries [6].

While worldwide wasting in infants and young children is decreasing, Africa estimates that 10% of infants and young children are moderate to severely wasted [7]. Despite Ethiopia's initiatives to fight poverty and food insecurity, many rural areas are still exposed to food insecurity and wasting due to seasonal factors [8, 9]. According to a study conducted in the southern region of Ethiopia, wasting affects 14.6% of infants and young children [10]. A review and meta analysis conducted in Ethiopia estimated that the prevalence of wasting among infants and young children was 15% [11]. Wasting has also been observed to be prevalent (16.2%) among infants and young children in the Afar reginal state of Ethiopia [12]. Furthermore, a wasting prevalence of 7% was observed in the Ethiopian Mini Demographic and Health Survey in 2016 [13].

Several Ethiopian study findings have found that socioeconomic and demographic variables influence the prevalence of wasting among infants and young children [14, 15]. Infant and young child wasting is linked to poor food intake, housing, and water quality [14]. Moreover, birth order [15, 16], a lack of screening [17, 18], and diarrhoea [12, 19–21] have all been linked to wasting. The gender of infants and young children and their age are characterized as variables that influence wasting [17, 22, 23]. Wasting is also linked to educational status [24, 25], occupational status [26], family food insufficiency [27, 28], and dietary intake [21, 29, 30].

Furthermore, the nutritional condition of the parents [6] and the family socioeconomic status [17, 31, 32] are the most important factors related to wasting among infants and young children in low- and middle-income countries. In Ethiopia, the number of children under the age of five, the duration of nursing, and the age at which supplemental feeding began were all significant variables associated with wasting. [33]. According to previous studies conducted, family size is a significant factor related to wasting among childhood [24, 27, 29].

Despite the fact that Oromia is one of Ethiopia's food-producing areas, the frequency of wasting among infants and young children were found to be significant at 6.9% [33]. Infants and young children from food-insecure regions have a significant prevalence (27%) of this condition [34]. As a result, Ethiopia's government works to improve the country's socioeconomic condition; however, socioeconomic variables and wasting are more complicated [35].

According to the Ministry of Labor and Social Affairs, the Productive Safety Net Program (PSNP) of a country is intended to eliminate poverty and bridge the food gap for vulnerable areas, and it encompasses all food security measures within the social protection policy [36]. Despite the fact that the program incorporates a variety of strategies to minimize food insecurity and enhance the nutritional health of infants and young children in the region, it has not yet reached its full potential due to disparities in resource distribution among communities.

The following are the reasons why the Kuyu district was chosen as the study area: (1) Kuyu district is known across the district for its heavy rainfall, low agricultural production, and low soil fertility and has received food assistance and food shortages from the PSNP for many years [37]. (2) The Kuyu district has a higher proportion of food-insecure rural residents who rely on the Productivity Safety Net Program for food or cash in exchange for labor [38]. (3) Several previous cross-sectional studies encompassed all potential food security locations and districts that did not require food assistance from the government or nongovernmental organizations. (4) Previous research findings from various locations and districts in Ethiopia were outdated, and they may no longer reflect the current state of wasting and related variables among infants and young children in the study area. (5) This research was conducted in a rural setting, where many rural households in the study area have been experiencing food insecurity and malnutrition for more than a decade. (6) In the study area, no research into the scope of wasting and its associated factors has been conducted to aid the most vulnerable group of people: infants and young children.

Thus, the findings of this study would bring up-to-date information on the nutritional status of infants and young children in the district's most food-insecure area. Taking the aforementioned rationales into mind, this study was therefore carried out in the Kuyu district of northern Oromia, Ethiopia, to assess the prevalence of wasting and related factors among infants and young children aged 6-23 months.

## 2. Material and Methods

### 2.1. Study Setup, Design, and Duration

The Kuyu district was chosen as a research site because it includes more food-insecure rural people who rely on the Productivity Safety Net Program for assistance. As a result, this community-based observational study was undertaken from July 12 to July 28, 2020, following the techniques of prior investigations [39]. The baseline population was all 6-23-month infants and young children found in the Kuyu district, while the study population was all 6-23-month infants and young children selected from the specified Kebeles. 6-23-month infants and young children and a mother from Kebele were involved in the research. The study excluded infants and young children less than six and above 23 months as well as with birth abnormalities, chronic diseases, and mothers who did not want to participate.

### 2.2. Determination of the Sample Size and Procedure

The following assumptions were made; 95% CI, 80% performance, *P*1 = 0.18; poor eating habits in children under 5 years [33] and 10% expected good eating habits in children under 5 years (*P*2 = 0.08). Therefore, the sample size was 392, the nonresponse rate was 5%, and the design effect was 612.

The Kuyu district area was carefully chosen as the research location since previous studies had not investigated the prevalence and critical characteristics related to wasting in infants and young children aged 6-23 months. As a result, the findings of this study can help Ethiopians with nutrition and nutrition-sensitive agricultural policy. In this study, a multilevel sampling method was used. Using the size-proportional likelihood technique, four Kebeles (Sombo Cheka, Halilu Cheri, Dubena Agalo, and Wuyye Gose) were chosen for the research among the 20 district Kebeles. The district health department gathered data on infants and young children aged 6-23 months. In four Kebeles households (Sombo Cheka, Halilu Cheri, Dubena Agalo, and Wuyye Gose), the total number of infants and young children aged 6-23 months was 448, 712, 775, and 865, respectively. Then, in Kebele, the method of selecting a 6-23-month infant and young child from each household was chosen. Finally, each Kebele infant and young child were chosen at random from each category's list of households. If a household had more than one mother with infants and young children aged 6-23 months, only one mother was chosen by lot, and the same procedure was used if the household had more than one infant and young child who met the selection criteria.

### 2.3. Data Collection Methods and Quality Assurance

Wealth index, age of the infant and young child and mother, sex of the infant and young child, head of household, size of family in household, occupation, level of education, and ethnicity were all surveyed sociodemographic data. The children's weight and height were measured according to WHO guidelines [40]. A local event was used to compute the child's age in months from the date of birth to the date of data collection. Moderately pressing both feet for 3 seconds was also used to detect edema. The data collector consulted the supervisor for confirmation, and a referral to the nearest medical facility if the depression remained flat on both feet for a few seconds.

To achieve the study's main goals and reduce bias during data collection, the following measures were considered: first, data were collected using a structured questionnaire adapted from related studies. The questionnaire was written in English and then translated into a local language (Afaan Oromoo) with few changes based on previous research. It was then checked for consistency by having it translated into English by experts in various languages. The survey was then pretested on 5% of the sample before we started collecting data. We made the necessary corrections and changes to the terms and format of the questionnaire based on the feedback. Third, data was gathered from 10 registered nurses and three public health/nutrition specialists and researchers after a three-day training session for data collectors and supervisors. The principal investigator in charge of the study double-checked the questionnaire's accuracy at the end of each day.

### 2.4. Data Analysis

SPSS version 20.0 was used to encode, enter, and analyze the data. All variables were subjected to descriptive statistical analysis to look for outliers, data consistency, and missing values. A one-sample Kolmogorov-Smirnov test was used to check the normality of continuous variables. The WHO Anthro program version 3.2.2 was used to generate infant and young child height and weight from WHO growth standards. If the *z*-scores for each index were less than 2, the child was considered wasted. At a *P* value of 0.05, a logistic regression analysis was used to identify the factor linked to wasting. Finally, AOR was calculated at a 95% confidence level.

### 2.5. Ethics and Consent

The Wollega University Food and Nutritional Sciences Institutional Review Board Committee (IRBC) provided ethical approval with Ref No. WuIRBC-0789/2020. The study's purpose was communicated to officials from the Kuyu City Public Health Administration, who granted approval and assistance. All study participants were informed about the study's purpose, and written informed consent was obtained. The responses were coded to keep them private. Finally, the mothers and infants and young children with severe wasting received nutritional and health information in preparation for further treatment.

## 3. Results

### 3.1. Sociodemographic Characteristics of Survey Participants

The Oromo ethnic group was represented by 604 mothers (98.7%). About 490 (80.1%) and 304 (49.7%) of the participants were married and illiterate, respectively (Table 1). Moreover, half of the mothers (51.6%), were farmers. Two-thirds of the participants (67.5%) had a family of more than five members. In addition, 326 (53.3%), 163 (26.6%), and 123 (20.1%) households were classed as having low, medium, or high wealth index, respectively.

### 3.2. Child Characteristics

About 30.6% of children are born at home, while 69.4% are born in hospitals. Almost half of the infants and young children (48.2%) were not immunized (Table 2). In addition, 17.3% and 7.7% of the infants and young children suffered diarrhoea and edema, respectively.

### 3.3. Child Feeding and Caring Characteristics

According to the findings, about 209 (34.2%) mothers began nursing within one hour, and 403 (65.8%) mothers began breastfeeding one day later (Table 3). More than half of the 612 mothers (64.2%) did not feed their infants and young children. Milk is given to infants before colostrum feeding, which accounts for 86.6% of the time. Furthermore, two-thirds (65%) of the mothers did not just breastfeed their infants and young children but also fed them other meals. Approximately 43% and 68.9% of infants and young children, respectively, had less than recommended nutritional diversity and meal frequency (Table 3).

### 3.4. Maternal Characteristics

In this study, 174 (28.4%) mothers gave birth to their first child before the age of 18 (Table 4). The proportion of mothers who did not take part in the check-ups was 68.9%. The majority of mothers who participated in this study were unaware of their children's eating habits (74.2%).

### 3.5. Environmental Condition

The majority of mothers in the study area (79.6%) used unprotected drinking water (Table 5). Of the 612 mothers, 80.9% and 57.2%, respectively, had no toilet or separate kitchen. In addition, 234 (38.2%) mothers used open land for waste disposal.

### 3.6. Prevalence of Wasting

The current study showed that the prevalence of wasting among infants and young children aged 6-23 months in the study area was 14.1% (Table 6).

### 3.7. Selected Associated Factors of Wasting

Multivariate analysis revealed that maternal upbringing, breastfeeding, antenatal visits, and wealth index are factors associated with child wasting in the study area (Table 7). The results showed that those infants and young children from illiterate mothers (AOR = 1.8; 95% CI, 1.01.4.32), who had diarrhoea (AOR = 2.3; 95% CI, 1.98-4.56), and who had lack of exclusive breastfeeding (AOR = 2.46; 95% CI, 1.4-4, 58) more were wasted than that of the reference. Similarly, the odds ratio for infant and young child wasting was higher in mothers who did not attend antenatal care visits (AOR = 2.21; 95% CI, 1.32-3.48) and had low wealth status (AOR = 1.66; 95% CI, 1.07-4.47).

## 4. Discussion

According to the findings of this study, the prevalence of infant and young child wasting in the study area was greater than in Ethiopia [41–43]. Other investigations conducted in Pakistan [20] and Ethiopia [22, 23, 44] found it to be lower. Differences in the quality of treatment, the duration of data collection, the disciplines of study, and socioeconomic inequalities in the field of study might all be factors in this disparity.

Children born from illiterate mothers were 1.8 times more likely to have wasting than those infants and young children from educated mothers. This finding was supported by research from Ethiopia [23, 44] and Burkina Faso [45]. This might be because informed women are better able to comprehend nutrition and health information, allowing them to enhance their infant's and children's nutritional status. Infants and young children who had diarrhoea throughout the trial were 2.3 times more likely to be wasted than those who did not have diarrhoea. This conclusion was supported by research from Burkina Faso [45] and Ethiopia [20, 46]. This might be due to the fact that diarrhoea is a direct cause of the child's nutritional issues.

In this study, nonbreastfed infants and young children were 2.46 times more likely to be wasted than breastfed. Other investigations conducted in Nigeria [47] and Indonesia [48] corroborated this finding. This is assumed to be due to the fact that breastfeeding delivers all of the nutrients required for appropriate growth and intellectual development, which might have an influence on a child's health and nutrition. Furthermore, mothers who did not get antenatal check-ups (ANC) had 2.21 times the number of wasted infants and young children than those mothers who did it. The findings of this investigation were similar to those reported in Ethiopia [17] and India [19]. This might be due to the fact that ANC visits serve to reduce threats to a child's health and nutritional condition.

According to a multivariate analysis of this study, infants and young children from low-income families are 1.66 times more likely to be wasted than infants and young children from high-income families. These findings are in line with previous studies [49, 50]. Similar findings have been found in Ethiopia, suggesting that low socioeconomic level is a role in the accumulation of garbage [32]. This might be because low-income families are unable to provide a healthy diet for their infants and young children due to budgetary constraints.

### 4.1. Limitations of the Study

Because the study was done over a single time period, it is possible that the real nutritional status of infants and early children was not captured. It was also cross-sectional research; therefore, no cause-and-effect link between the predictors and the outcome variables could be established. The outcomes of this study might be influenced by recall bias during the interview and anthropometric measurement problems.

### 4.2. Implication of the Study

This study was a community-based approach, in which study subjects were randomly selected from the targeted population. The sample size was calculated using a single population formula. This could be representative and may be made possible generalization to the target communities in the study area. Moreover, a pretest (5%) was conducted before the actual data collection began.

## 5. Conclusion

The current study found that the frequency of wasting among infants and young children aged 6-23 months was significant in the Kuyu area of central Oromia, Ethiopia. According to this study, the key indicators linked to infants and young children wasting include maternal/caregiver educational status, diarrhoea, exclusive breastfeeding, prenatal visits, and wealth index. Therefore, nutrition and health-based education should be encouraged in order to enhance awareness and minimize the problem of wasting among infants and young children and improve household economic status.

## Figures and Tables

**Table 1:** Socioeconomic and demographic characteristics.

Variables	Frequency (no.)	Percent (%)
Age of the mothers (years)	65	10.62
≤24	130	21.24
25-29	417	68.14
≥30		
The educational level of respondent		
Illiterate	304	49.7
Able to read and write	126	20.6
Elementary school and above	182	29.7
Marital status of the respondent		
Married	490	80.1
Divorced	53	8.7
Others (single, widowed)	69	11.3
Occupational status of the respondent		
Housewife only	91	14.9
Farmer	316	51.6
Others (merchant, daily laborer)	205	33.5
Ethnicity of respondent		
Oromo	604	98.7
Others (Amhara, Tigre)	8	1.3
Family size in the household		
<5	199	32.5
≥5	413	67.5
Wealth index		
Low	326	53.3
Middle	163	26.6
High	123	20.1

**Table 2:** Child characteristics.

Variables	Frequency (no.)	Percent (%)
Sex of the study child		
Male	324	52.9
Female	288	47.1
Age of the child		
6-12	406	66.3
13-23	206	33.7
Place of delivery		
Home	187	30.6
Health institution	425	69.4
Immunization		
Yes	317	51.8
No	295	48.2
Diarrhoea		
Yes	106	17.3
No	506	82.7
Edema		
Yes	47	7.7
No	565	92.3

**Table 3:** Child feeding and caring characteristics.

Variables	Frequency (no.)	Percent (%)
Time of breastfeeding		
Within one hour	209	34.2
After one day	403	65.8
Colostrum's given		
Yes	219	35.8
No	393	64.2
Pre-lactation food given		
Milk	530	86.6
Butter	69	11.3
Water	13	2.1
Exclusively breastfeeding		
<6 months	398	65
≥6 months	214	35
Complementary feeding		
Before six months	311	50.8
At six months	95	15.5
After months	206	33.7
Dietary diversity		
<3	263	43
≥4	349	57
Child meal frequency		
≥4	191	31.1
≤3	421	68.9

**Table 4:** Maternal characteristics.

Variables	Frequency (no.)	Percent (%)
Age at first birth (in years)		
<18	174	28.4
18-28	438	71.6
Antenatal care visits		
Yes	191	31.1
No	421	68.9
Knowledge about feeding practices		
Yes	158	25.8
No	454	74.2
Hand washing materials		
Soap	213	34.8
Water only	399	65.2

**Table 5:** Environmental condition.

Variables	Frequency (no.)	Percent (%)
Source of drinking water		
Protected	125	20.4
Unprotected	487	79.6
Presence of latrine		
Yes	117	19.1
No	495	80.9
Separate kitchen		
Yes	262	42.8
No	350	57.2
Solid waste disposal		
Open	234	38.2
Private	173	28.3
Common	205	33.5

**Table 6:** Prevalence of wasting.

Undernutrition (wasting)	Frequency (no.)	Percent (%)
Normal	526	85.9
Wasted	86	14.1

**Table 7:** Selected associated factors of wasting.

Variables	Odds ratio	
	COR (95% CI)	AOR (95% CI)
Mother's educational status		
Illiterate	2.1 (1.9-7.4)^∗^	1.8 (1.01-4.32)^∗∗^
Able to read and write	1.2 (1.3-5.42)^∗^	1.23 (0.65-3.12)
Elementary school and above	1.0	1.0
Diarrhoea		
Yes	1.24 (2.3-11.1)^∗^	2.3 (1.98-4.56)^∗∗^
No	1.0	1.0
Exclusively breastfeeding		
Yes	1.0	1.0
No	1.85 (1.04-3.67)^∗^	2.46 (1.40-4.58)^∗∗^
Antenatal care visits		
Yes	1.0	1.0
No	1.26 (1.25-1.93)^∗^	2.21 (1.32-3.48)^∗∗^
Wealth index		
High	1.0	1.0
Middle	1.04 (1.05-2.14)^∗^	1.12 (0.98-3.45)
Low	1.40 (1.02-3.81)^∗^	1.66 (1.07-4.47)^∗∗^

^∗^ *P* value < 0.25 in the bivariate analysis and ^∗∗^*P* value < 0.05 in the multivariate analysis and 1 = References.

## Data Availability

Data to support the findings of this study is available on reasonable request from the corresponding author.
